The article "Green human resources management: A novel tool to boost work engagement" was published in 2022. Journal: Front Psychol.

# Green human resources management: A novel tool to boost work engagement

**DOI:** 10.3389/fpsyg.2022.951963

**Published:** 2022-10-25

**Authors:** Elif Baykal, Osman Bayraktar

**Affiliations:** ^1^Business Administration Department, Istanbul Medipol University, Istanbul, Turkey; ^2^Business Administration Department, Istanbul Commerce University, Istanbul, Turkey

**Keywords:** human resource management, social sustainability, green human resources management, psychological ownership, work engagement

## Abstract

Increasing environmental awareness in business life has given way to Green Human Resources Management practices. The positive corporate image created by GHRM is encouraging for many employees and boosts their work engagement. GHRM practices make employees feel proud about their organization and creates a value-based ground for working in their current companies. Actually, internalized green inclinations of organizations, namely, value alignment between an organization and an employee, can make their employees feel greater psychological ownership about their companies, leading to greater engagement as it is suggested in social identity theory. Being inspired from psychological ownership literature, in this study, it is assumed that being exposed to Green Human Resources Management practices can make employees feel higher levels of work engagement and psychological ownership can have a mediator effect in this relationship. The model has been a tested model among 255 Turkish white-collar employees working in a manufacturing sector. Analyses have been carried out using the AMOS structural equation program and the PROCESS program. Results confirmed the above assumptions, confirming the assumptions of social identity theory and revealed the existence of mediator effect in the relationship between GHRM and work engagement of employees, illuminating the importance of GHRM for employees' positive attitudes toward their organization.

## Introduction

The growing awareness about environmental sustainability has given way to the concept of green human resource management. Ren et al. (2017) explained this novel HRM approach as a “phenomenon relevant to understanding relationships between organizational activities that impact the natural environment and the design, evolution, implementation, and influence of HRM systems. GHRM encompasses implications regarding hiring and retaining environmentally friendly employees and ways to retain them (Susanto et al., 2022). Moreover, in order to talk about a strong GHRM department, organizations should implement proper training programs, rewards, and benefits systems (Mishra, 2017). That is to say, GHRM practices facilitate the application of green practices through different practices, such as recruitment and selection, wage management, performance management, and exit policies (Nisar et al., 2021).

The importance of GHRM stems from the fact that it is a critical component of an environment-oriented strategic plan to build, maintain, and strengthen sustainable development (Farooq et al., 2021). Companies proactively engaging in GHRM can create a “green” image, and this green image can prevent negative impacts of adverse events. Actually, GHRM practices can be accepted as predictors of green environmental performance impacting a supply chain: production, culture, strategies, and even employee behaviors (Benevene and Buonomo, 2020).

GHRM creates a positive employer brand for a company leading to many positive organizational outcomes, including work engagement. In this context, work engagement should be understood as physical and psychological conditions related to work cognitively and emotionally, encouraging attitudes and behaviors necessary for achieving organizational level goals (Keyko et al., 2016). Emotional attachment with a target of possession can positively affect employees' attitudes in an organization and result in higher levels of identification and engagement (Schaufeli et al., 2017), and it can create advantage for organizations on their journey for sustainability by making employees prefer to stay in their organization and work hard for its strategic goals (Carmeli et al., 2022). As to Chang et al. (2020), a common vision regarding an organization's green intiatives conveyed through GHRM can promote sustainable development, and this can strengthen employees' feelings of psychological ownership. Hence, in this study, we assumed that employees embrace green tendencies of their organizations and feel greater ownership on their organizations leading to higher levels of engagement. Unfortunately, in the extant literature, there is a scarcity of research examining the role played by GHRM in enhancing psychological ownership and work engagement. Previous studies on GHRM-work engagement relationship (Aktar and Islam, 2019; Aboramadan, 2020; Darban et al., 2022) revealed a direct effect of GHRM on work engagement. On the one hand, many other studies revealed that, as an organizational outcome, work engagement is possible mostly through feelings of psychological ownership (Rapti et al., 2017; Su and Ng, 2019; Wang et al., 2019), which makes psychological ownership worth examining in the relationship between GHRM and work engagement.

In this point, social identity theory, explaining that individuals tend to attach their possessions, is illuminating in revealing the positive effect of psychological ownership on engagement (Narcikara, 2017). Cognizant of the need to better understand the impact of GHRM practices on work engagement, in this study, it is aimed to illuminate the possible effect of GHRM on work engagement levels of employees and the possible mediator effect of psychological ownership in the relationship between GHRM and work engagement. Hence, the research question of the study is explanatory about psychological ownership's mediator effect in the possible positive effect of GHRM on work engagement. GHRM studies are still infertile in HRM literature despite its importance regarding sustainability and employee engagement (Malik et al., 2021; Qadri et al., 2022). In previous studies, although there are a considerable number of studies revealing the positive effect of HRM on psychological ownership (Masnita et al., 2019) and on work engagement (Shantz et al., 2016; Sousa et al., 2021), there is not any study explaining the above-mentioned relationships in relation to GHRM. Moreover, it is seen that there is no previous study about the possible mediator effect of Psychological Ownership in the relationship between HRM/GHRM and work engagement. Hence, as a considerable contribution to GHRM literature, the relationship between GHRM, psychological ownership, and work engagement, which has been identified as a gap, will be clarified. In addition, as a managerial output, it is anticipated that findings of this study can encourage the use of GHRM as a human resources tool of ensuring work engagement and retention of employees contributing to a greater possibility for sustainable organizations. This study was conducted especially in the Turkish production sector, since this sector is the one that needs environmentally friendly activities most. Moreover. it is the most noteworthy sector in that it is the sector that has the biggest potential to threaten the environment. Therefore, it is thought that an environmentally conscious HRM structuring in the production sector will make a greater contribution to the stakeholders, especially to the employees, and will increase their work engagement.

## Theoretical background and development of hypotheses

The green performance of companies is an emerging issue, gaining greater importance on the agenda of global corporations (Guerci et al., 2016), and GHRM research has become popular after 2011 (Paulet et al., 2021). As to Ren et al. (2017), the alignment of human resources management practices with an organization's green policies creates ‘Green Human Resources Management'. GHRM research is explained as the HRM aspects of environmental management (Renwick et al., 2013). It is those parts of sustainable human resources management dealing with specifically environmental sustainability (Wagner, 2013).

According to Ren et al. (2017), for providing environmental awareness, employees are the key to success. The basic requirement of GHRM is empowering workers so that they can make recommendations that are effective for contributing to the environment (Ali et al., 2020). GHRM motivates employees by rewarding their green performance and by stimulating employees' involvement by empowering them and creating an environmentally friendly climate (Aboramadan, 2020; Ansari et al., 2021). It is concerned with changing ordinary employees into green employees so that they can help their organizations in green issues (Arulrajah et al., 2015; Jermsittiparsert, 2021) and in this transition, the sense of ownership and engagement are important. GHRM practices develop green abilities through HR activities like green recruitment, selection, performance management, and training. For example, Green recruitment and selection try to attract employees with green awareness (Tang et al., 2018), whereas green training attempts to change attitudes and emotional involvement toward green organizational goals (Zibarras and Coan, 2015) and green performance management reward pro-environmental contribution of employees (Úbeda-García et al., 2021).

GHRM lowers absenteeism and turnover levels (Al-Hajri, 2020; Darban et al., 2022) and organizational commitment (Shoaib et al., 2021) and contributes to work engagement (Aktar and Islam, 2019; Alshaabani et al., 2021). Actually, work engagement is a dynamic cognitive and emotional dimension, explaining personal enthusiasm about one's work (Wu et al., 2022). In this study, it is believed that studying work engagement is significant since it contributes to higher performance (Neuber et al., 2022; Yao et al., 2022) and intention to stay (Parent-Lamarche, 2022) that are necessary for applying GHRM. It is signified by energy, involvement, and self-efficacy (Chen et al., 2020). It is a positive emotional state related to work that should be explained in three main dimensions: vigor, dedication, and absorption (Schaufeli et al., 2006; Gómez-Salgado et al., 2021). Vigor explains high levels of energy and resilience at work; it is persistence in times of turmoil; dedication explains feelings of enthusiasm and importance; and absorption refers to being fully engrossed in one's work (Schaufeli et al., 2006). In fact, work engagement is a multiaxial concept effected by multiple factors including organizational climate, job resources, psychological resources, and sense of ownership (Keyko et al., 2016). Moreover, as Rollins et al. (2021) explain, a sensible work climate can boost employee work engagement.

In this study, we assumed that one possible antecedent of work engagement is psychological ownership. Psychological ownership is a psychologically felt phenomenon in which individuals develop a sense of ownership for a goal (Van Dyne and Pierce, 2004). It is the result of concentration, consideration, and deliberation on one's possessions (Jami et al., 2021). It helps individuals create and maintain their self-identity (Fritze et al., 2020). Antecedents of psychological ownership are perceived control, self-investment, and knowledge (Morewedge et al., 2021). With the help of psychological ownership, properties associated with the self are transferred to the target, thus increasing emotional attachment to the target and boosting its value (Weiss and Johar, 2016).

In this study, social identity theory and conservation of resources theory have been considered as a theoretical framework while building a hypothesis. Identification is anchored in social identity theory, and, in this theory, engagment is closely related with reasons creating social membership (Pierce et al., 2001). According to social identity theory, possessions serve as symbolic expressions of the identity, and they are closely connected with individuality; that is why individuals engage to an object and use this ownership for defining themselves and expressing their identity (Pierce et al., 2001). On the one hand, the sense of ownership creates the inclination to protect the possession; that is why employees identifying themselves with their organizations often make their best to continue their existence in their social groups and engage to their organizations (Narcikara, 2018). Similarly, conservation of resources theory claims that individuals have an innate tendency to protect their both tangible and intangible possessions like their membership in a group, their jobs, their friends, etc.; hence, people consider it charming to continue their existence in their social groups (Hobfoll et al., 2000).

In relation to the positive associations mentioned above, in this study, it is assumed that psychological ownership has the capacity to contribute to positive outcomes, such as motivation, satisfaction, engagement, high performance, and continuity, which are necessary for attaining organizational ends targeted by GHRM. Sense of ownership regarding an organization will make the employees stick strictly to its values and strategies (Maharani et al., 2021), which is significant for creating devoted employees to green issues and ensuring their sincere engagement to the company. The fact that the mediator effect of psychological ownership in the relationship between GHRM and work engagement has not studied in the extant literature, in this study, it is aimed to see whether the positive effect of GHRM on work engagement is possible through psychological ownership or not.

## Hypothesis

When we turn our lens to work engagement, it can be seen that myriad factors affect work engagement levels of employees. Motivation enhancing human resources practices (Amir et al., 2022; Beltrán-Martín et al., 2022) and value match between an individual and an organization (Okolie, 2022) are considered as significant antecedents of work engagement. According to social identity theory, when individuals work in an organization with responsible practices they are proud of, their identification with their organziation increases (Yang et al., 2021). In this sense, employees who think that the reputation of their institutions has increased due to GHRM will also feel greater social identification with their company, and this will increase their work engagement since they will enjoy being part of a highly reputable organization (Ahmad et al., 2022). In the extant literature, we can come across considerable number of empirical proofs revealing the positive impact of socially responsible human resources management practices on employee work engagement supports this view (Abid et al., 2018; Gürlek and Tuna, 2019). In relation to GHRM-work engagement relationship, there are also empirical pieces of evidence inspiring our first hypothesis. For instance, Aboramadan (2020), Ababneh (2021), and Darban et al. (2022) proved the positive relationship between GHRM and work engagement. Hence, being inspired from the extant literature, it is assumed that, when individuals notice their organizations' socially responsible GHRM practices, their work engagement levels improve. So, it is hypothesized that:

H1: GHRM has a positive effect on work engagement.

On the one hand, as O'driscoll et al. (2006) suggest, sensible and responsive business environments lead to the development of psychological ownership since increased control over the target gives the opportunity to better know and focus on the target. Similarly, Appelbaum et al. (2000) suggest that HRM practices that promote abilities, motivation, and opportunities of individuals and create a responsible organizational climate can contribute to psychological ownership feelings of employees. Anyway, in the related literature, it has been revealed that GHRM leads to a sensible organizational climate, leading to organizational commitment that gives birth to psychological ownership in the long run (Pham et al., 2019). As it is explained in conservation of resources theory, individuals tend to attach to their possessions when they are committed to them (Zhang et al., 2021). Besides that, in previous studies, traces for the positive effect of human resources practices on psychological ownership can be found that encouraged us for studying the same effect regarding GHRM. For instance, Mayhew et al. (2007) signified that many human resources-related factors, including job design and autonomy, affect psychological ownership perceptions of employees. Later, Degbey et al. (2021) and Waqas et al. (2021) confirmed that HRM practices have the potential to affect psychological ownership feelings of employees. In relation to GHRM, Chang et al. (2020) also revealed the positive effects of green values in an organizational climate that can be created by GHRM on psychological ownership feelings of employees. Being inspired by the extant literature, we assumed that GHRM practices will also have a positive impact on employee psychological ownership. Hence, it is hypothesized that:

H2: GHRM has a positive effect on psychological ownership of employees.

The basic tenet of conservation of resources theory is that people try to retain and protect those things that they value (Hobfoll et al., 2000). Interestingly, this is a mutual relationship since, when individuals develop a sense of ownership, they also build an emotional attachment with the target, and this increases their engagement with the target (Morewedge, 2021). Similarly, when employees build a sense of ownership regarding their organizations, they will become emotionally attached to their organization, and this will build higher levels of work engagement (Baker et al., 2021). According to the Resource Investment principle of conservation of resources theory, individuals invest in resources to prevent the loss of them (Zhou and Chen, 2021). Considering this fact, in this study, it is assumed that, when employees have a sense of ownership regarding their organizations, they would prefer continuing to be a part of these organizations and working hard with enthusiasm and engagement in order not to lose their membership. In this point, there are empirical proofs revealing this positive relationship. For example, Su and Ng (2019) revealed a positive effect of psychological ownership on work engagement among social workers. Wang et al. (2019) confirmed the same relationship in the Chinese context. Later, Sokro et al. (2020) confirmed the same relationship empirically. Similarly, Khan and Gul (2021) revealed the positive effect of psychological ownership on work engagement and revealed the mediating role of work engagement in the relationship between psychological ownership and happiness. In addition, Nurtjahjani et al. (2021) also confirmed that the higher the employees' belief in a just world in their organizations, the stronger the relationship between psychological ownership and work engagement. Being inspired by these studies, it is hypothesized that psychological ownership will have a positive effect on work engagement. Thus, the following hypothesis has been built:

H3: Psychological ownership has a positive effect on work engagement.

According to Primary Loss Principle of Conservation of Resources theory, the effect of resource loss is greater than resource gain (Zhou and Chen, 2021). Hence, employees would not want to lose the comfort and satisfaction of working in a sensible, stakeholder-friendly positive climate. For many individuals, being exposed to GHRM can boost their Psychological Ownership feelings, and this can mediate the effect of GHRM on work engagement, owing to primary effect. In the related literature, although there is no similar previous study showing the effect of GHRM practices on work engagement through psychological ownership, there are some previous studies showing the positive effect of human resources practices, in general, on work engagement through the mediator effect of psychological ownership. In this sense, in the research conducted by Duran (2019), it was determined that psychological ownership has a mediating effect on the positive effect of human resources practices on work engagement. Similarly, Olckers and Du Plessis (2012) revealed the mediator role of psychological ownership in retaining and engaging talent in HRM's effect on engagement and intention to stay, and, later, being inspired from these studies, we assumed that psychological ownership can have the same mediator effect on the relationship between GHRM and work engagement. Thus, we hypothesized that:

H4: Psychological ownership mediates the relationship between GHRM and work engagement.

### Research design

The purpose of this research is to test the mediating role of psychological ownership in the relationship between GHRM and work engagement. In the research model, GRHM was included as an independent, work-related, psychological ownership tool variable. It is aimed to collect the research data from white-collar employees operating in the production sector in Istanbul. It is aimed to reach people working in the automotive, chemical, and food sub-sectors within the production sector. The manufacturing sector is specifically chosen fort the study since green issues are more important in this sector in relation to tangible production and greater possibility of affecting the environment.

As it is shown in Figure 1, the research model describes the relationship between green human resources management practices (GHRM), psychological ownership (PO), and work engagement (WE).

**Figure 1:** The research model.

## Materials and methods

### Samples and procedures

Both the face-to-face survey method and the online survey method were used to collect data for this study. Face-to-face surveys have been carried out in companies that allow the application of the survey during work hours, whereas online surveys have been collected through social media portals mostly *via* LinkedIn. The accounts of 30 thousand professionals were examined, and an online questionnaire was sent to the profiles suitable for the sample of our research. The constructs in our study were developed using measurement scales adopted from previous studies. Survey items were responded with five-point Likert scales, with anchors ranging from strongly disagree (1) to strongly agree (5). We used a convenience sampling method to collect our data. Convenience sampling has been preferred, owing to time and budget restrictions in this study. Approximately, 320 surveys have been delivered to people working in Istanbul using the face–to-face survey method. Moreover, 540 surveys were disseminated *via* an Internet survey program to reach applicants working with the teleworking model. Approximately, 260 people (83%) answered our questionnaire. The forms of 10 participants were excluded from the evaluation, and 255 forms were analyzed.

We distributed our surveys between October 2021 and November 2021. Participation from companies employing 50 or less people was not taken into account while collecting data. In Turkey, Istanbul is the main business center, and nearly all corporate manufacturing firms are located in Istanbul, which directed our choice about sampling.

Since it is difficult to estimate the number of people in the research population, significant absolute values were used for statistical analysis in determining the sample size. There are different approaches among scientists based on the number of variables in determining the sample size. While some scientists advocate having 10 times as many participants as the number of variables, some scientists consider five or at least 100 participants per variable sufficient (Sencan, 2005, p. 362). The sample size of 200 people is considered sufficient for reliable factor analysis (Çokluk et al., 2018, p. 206). As a general rule, confirmatory factor analysis and SEM analysis are not considered appropriate for data below 150 (Müller, 2003; Gürbüz, 2019, p. 30). Based on these assumptions, it was aimed to reach > 200 samples in data collection. Details of the participants are shown in Table 1.

**Table 1:** Sample characteristics.

**Measure**		**Frequency**	**Percent**
Age	20–29	86	34.4
	30–39	95	38
	51–59	56	22.4
	60+	2	0.8
Gender	Male	122	48.8
	Female	128	51.2
Position	Top manager	33	13.2
	Middle manager	75	30
	HR manager	8	26.8
	Sub manager	67	3.2
	HR stuff	30	12
	Consultant	23	9.2
	Other	12	4.8
	Missing	2	,8
Seniority	0–2 year	71	28.4
	3–5 year	73	29.2
	6–10 year	44	17.6
	11–20 year	43	17.2
	21+ year	19	7.6
Marital status	Married	143	57.2
	Single	107	42.8
Emoloyee number in company	51–250	32	12.8
	251–500	21	8.4
	501–1,000	32	12.8
	1,000+	165	66
Sector	Automotive	104	41.6
	Chemistry	60	24
	Food	86	34.4

### Measurement tools

#### GHRM scale

Green human resources management (GHRM) was measured by a 20-item GHRM scale developed by Shah (2019) and adapted to Turkish by Öselmis (2020). This scale involves five sub-dimensions: green job design (4 items), green recruitment and selection (4 items), green training and development (3 items), green performance appraisal (4 items), and green wage management (5 items). On a 5-point Likert-type scale, the respondents indicated how strongly they agreed or disagreed with each topic (1 = strongly agree, 5 = strongly disagree). Considering the results of exploratory factor analysis, the scale was used as one-dimensional construct in this study (see Table 1). Before deciding on the GHRM scale, Tang et al. (2018) and Cabral and Dhar's (2019) scales were examined. Cabral and Dhar's scale is for collecting qualitative data. Since the questionnaire method was preferred in data collection and the participants were Turkish-speaking people, it was preferred to use a scale whose validity and reliability studies were conducted in Turkish. The scale used in the research is very similar to the scale developed by Tang et al. (2018).

#### Work engagement scale

To measure work engagement, short version of a Utrecht (UWES-3) work engagement scale developed by Schaufeli et al. (2009) has been used. On a 5-point Likert-type scale, the respondents indicated how strongly they agreed or disagreed with each topic (1 = strongly agree, 5 = strongly disagree; see Table 2). The Turkish adaptation of the short version of the 6-item Utrech scale was made by Güler et al. (2019).

**Table 2:** Factor loadings.

**Construct**		**Items**	**Standardized factor loadings**			**Scale reliability**
			**EFA**	**CFA1**	**CFA2**	
Green job design	1	My company has assigned various responsibilities related to environmental protection to each position in the organization.	0.805	0.802	0.868	Cronbach α; 0.935
	2	The company has included the green and social needs of the institution in its job descriptions and specifications.	0.847	0.845	0.923	SCR= 0.945
	3	My company includes green capabilities as a prominent element in its job specifications.	0.871	0.868	0.938	AVE= 0.812
Green selection and training	4	My company designs and implements innovative job positions to demonstrate the importance of environmental protection issues.	0.841	0.844	0.884	Cronbach α; 0.963
	5	Our company includes the criterion of “green awareness (Environmental Awareness)” in its human resources employment policies.	0.879	0.887	0.915	SCR= 0.951
	6	Our organization attracts candidates who attach importance to applying green criteria in order to create a green employer brand.	0.899	0.906	0.952	AVE= 0.867
	7	My company has a communication environment that enables the dissemination of green knowledge. skills and goals.	0.881	0.888	0.906	
	8	My company identifies who needs training in environmental management.	0.858	0.858	0.878	
	10	My company uses environmental protection elements as the main themes of green education.	0.897	0.901	0.936	
	11	My organization provides environmental management training to improve the awareness. skills and knowledge of employees on environmental management.	0.877	0.882	0.904	
Green performance management	12	Our company sets green goals. objectives and tasks for each employee throughout the organization.	0.894	0.894	0.913	Cronbach α; 0.949
	13	Green criteria are used to evaluate employee performance in my company.	0.875	0.863	0.910	SCR= 0.942
	14	My company monitors whether the green targets are being met and whether the green targets are being met.	0.900	0.889	0.939	AVE= 0.0.825
Green wage management	16	Our compensation system recognizes and rewards contributions to environmental protection.	0.794	0.758	0.910	Cronbach α; 0.950
	17	My company rewards green skill acquisition.	0.844	0.810	0.968	SCR= 0.951
	18	My company rewards participation in green education programs.	0.824	0.787	0.958	AVE= 0.796
	19	My company rewards contributions to environmental management through non-monetary rewards such as paid leave. special leave. gifts to employees and their families.	0.751	0.712	0.850	
	20	My company recognizes employees' green initiatives by promoting and praising them throughout the organization.	0.791	0.758	0.848	
Self identity	2	My workplace is indispensable to me.	0.828	0.879	0.834	Cronbach α; 0.88
	3	It gives me pleasure to be a member of this establishment.	0.807	0.837	0.839	SCR= 0.876
	4	I am proud to be associated with this establishment.	0.744	0.683	0.766	AVE= 0.514
	5	I think my workplace gives me dignity.	0.822	0.757	0.710	
Protect focus	8	I thought that I have to warn employees who have harmful behavior to our workplace.	0.810	0.696	0.730	Cronbach α; 0.767
	9	I thought that if something goes wrong in our workplace, I have to prevent it	0.777	,870	0.864	SCR= 0.876
	10	I thought it is necessary to be informed to our supervisors about the negative situations in our workplace.	0.684	,648	0.661	AVE= 0.514
Internal responsibility	12	I am aware of what is expected of me for my workplace.	0.587	0.727	0.734	Cronbach α; 0.678
	14	It is important to me to fully meet the expectations of my workplace from me.	0.606	0.707	0.700	
Work engagement	1	At my work I feel bursting with energy.	0.836	0.776	0.743	Cronbach α; 0.43
	2	At my job. I feel strong and vigorous.	0.875	0.827	0.800	SCR= 0.853
	3	In am enthusiastic about my job.	0.857	0.819	0.862	AVE= 0.556
	4	My job inspires me.	0.850	0.824	0.881	
	5	I'am immersed in my work.	0.507	0.324	0.320	
Notes		(i) Principal Component Analysis with Varimax Rotation				
		(ii) KMO = 0.958. Bartlett Test; p < 0.001				
		(iii) Total Variance Explained (%); 71.915				
		(iv) All CFA Paths are statistically signifi cant at p < 0.001				
1st Order CFA		X2/df = 2.121. SRMR = 0.05. TLI = 0.934. CFI = 0.942. RMSEA = 0.067				
2nd Order CFA		X2/df = 2.305. SRMR = 0.06. TLI = 0.924. CFI = 0.930. RMSEA = 0.072				

#### Psychological ownership scale

Moreover, psychological ownership was measured through the scale developed by Uçar (2018). The 14-item scale includes four sub-dimensions, including self-identity (5 items), efficacy (2 items), protective focus (3 items), and internal responsibility (4 items). In this study, the scale was used as a one-dimensional construct in line with the exploratory factor analysis result (see Table 3). Three scales related to psychological ownership (Olckers, 2013; Shukla and Singh, 2015; Iseki et al., 2022) were examined, and the scale developed by Uçar (2018) was preferred because it was prepared in Turkish.

**Table 3:** Correlation matrix.

	**Construct**	**CR**	**AVE**	**1**	**2**	**3**	**4**	**5**	**6**	**7**	**8**
1	Job design	0.936	0.830	**0.911**							
2	Selection and training	0.963	0.814	0.913^***^	**0.902**						
3	Performance	0.942	0.845	0.840^***^	0.897^***^	**0.919**					
4	Wage man.	0.951	0.796	0.695^***^	0.759^***^	0.857^***^	**0.892**				
5	Work engagement	0.859	0.566	0.366^***^	0.345^***^	0.293^***^	0.182^**^	**0.752**			
6	Protect focus	0.786	0.554	0.216^**^	0.168*	0.121^†^	0.053	0.542^***^	**0.744**		
7	Self identity	0.870	0.628	0.562^***^	0.517^***^	0.497^***^	0.397^***^	0.630^***^	0.454^***^	**0.793**	
8	Internal resposibility	0.679	0.514	0.382^***^	0.352^***^	0.269^**^	0.225^**^	0.706^***^	0.728^***^	0.613^***^	**0.717**

*** Correlation is significant at the 0.001.

** Correlation is significant at the 0.01.

^**^Correlation is significant at the 0.05.

† P value smaller than 0.001. Bold values are expressing correlation values.

### Statistical analyzes

All statistical analyses were conducted using IBM SPSS 24 AMOS 24. The pragmatic approach is used to test the hypothesis. The current research performs descriptive analysis to assess the demographic characteristics of employees. Cronbach Alpha and CR (Comoposite/construct reliability) values are measured to calculate the internal consistency for all study variables. SPSS Amos was employed for construct validity analysis. Exploratory factor analysis (EFA) and confirmatory factor analysis (CFA) were conducted to see if the observed variables were theoretically loaded together and to evaluate construct, convergent, and discriminant validity and reliability values. The Pearson Bivariate Correlation is estimated for association among study variables. The research model was investigated using the Structural Equation Modeling technique. Hypotheses regarding the effect of the independent variable on the dependent variable and the mediating variable were tested using linear regression, and the hypotheses regarding the effect of the mediating variable on the independent variable were tested using multiple regression. To test the mediating role of psychological ownership between green human resources management practices and work engagement employed Model 4 of the Hayes PROCESS Procedure for SPSS Version.

Using principal component analysis with varimax rotation, an EFA was performed to see if the observed variables were loaded together as expected and were adequately correlated. In order to test the congruence of the data set, we performed a factor analysis using the Kaiser-Meyer-Olkin (KMO) sample sufficiency test and the Bartlett's test for equality of variances. As a result of the analysis, KMO was found to be 0.9658, which is above the desired level of 0.50, and the Bartlett's test was found to be at the 0.001 level of significance. Moreover, in anti-image correlation, matrix diagonal values were examined and proven to be above the desired level of 0.5.

Thus, it could be deduced that the sample data were appropriate for factor analysis. In exploratory factor analysis, the threshold for factor loadings was designated as 0.5 (Hair et al., 2014). In measuring the internal validity of factors, Cronbach's alpha values were computed; each Cronbach's alpha value was above 0.7. Thus, it was proven that there was internal validity between those factors, and inner validity of all factors was proven.

In order to validate the EFA results and analyze validity and reliability of measures, Maximum Likelihood method confirmatory factor analyses were applied. Moreover, modification indexes were investigated, and error values that had high modification values were covariated. In the end, fit indexes were found to be *X*^2^*/df* = 1.708, *SRMR* = 0.045, *CFI* = 0.962, *RMSEA* = 0.053. The confirmatory factor analysis results of the measurement model are shown in Figure 2.

**Figure 2:** The confirmatory analyses model. JD, Job design; STR, Selection and training; PER, Performance; PAY, Wage management; SI, Self identity; PF, Protective focus; IR, Internal responsibility; WE, Work engagement.

Because of the fact that, in this study, holistic effects of all sub-divisions of green human resources management and psychological ownership as a second-order factor analysis were conducted. Model fit indexes of this structure were found to be: *X*^2^*/df* = 1.981, *SRMR* = 0.092, *CFI* = 0.945, *RMSEA* = 0.063. As a result, it was concluded that fit indexes could be accepted as being in the desired level (Hu and Bentler, 1999). Furthermore, unidimensionality was ensured, owing to the fact that all factor loadings were above the desired level, and convergent validity and model fit indexes were at the desired levels (Anderson and Gerbing, 1988). First-level and second-level confirmatory factor analysis results regarding the variables in the measurement model are shown in Table 2.

Because of the fact that, in this study, holistic effects of all sub-divisions of green human resources management and psychological ownership as a second-order factor analysis were conducted. Model fit indexes of this structure were found to be: *X*^2^*/df* = 1.981, *SRMR* = 0.092, *CFI* = 0.945, *RMSEA* = 0.063. As a result, it was concluded that fit indexes could be accepted as being in the desired level (Hu and Bentler, 1999). Furthermore, unidimensionality was ensured, owing to the fact that all factor loadings were above the desired level and convergent validity, and model fit indexes were at the desired levels (Anderson and Gerbing, 1988). First-level and second-level confirmatory factor analysis results regarding the variables in the measurement model are shown in Table 2.

Furthermore, in order to test the reliability of factor structures, AVE (Average Variance Extracted) (Fornell and Larcker, 1981) and SCR (Scale Composite Reliability) values were used. When the AVE value is above 0.5 and when the CR value is above 0.7, it is proper to claim that related factors ensure validity and reliability (Bagozzi and Yi, 1988; Yaşlioglu, 2017). AVE and SCR values regarding the factors in this study are presented in Table 3. According to these values, our factors' validity and reliability are at the desired levels (see Table 3). Only the CR value of the internal responsibility dimension is slightly below the threshold value. It can be deduced that there is differential validity among factors (Hair et al., 2014).

## Results

### Findings related to the scales

#### GHRM scale

The original scale includes 20 items and five sub-dimensions: green job design, green selection, green education and development, green performance, and green wage management. As a result of the CFA analysis, items 9, 11, and 15 were removed from the scale because they were included in different dimensions. The items in the green selection and green education sub-dimensions were collected in a single factor, and the scale finally consisted of 17 items and four dimensions.

#### Psychological ownership scale

The original 14 item scale contains four sub-dimensions: self-identity, efficacy, protective focus, and internal responsibility. In the CFA analysis, the scale items were distributed in four dimensions as in the original. However, since the two-item efficacy scale, Cronbach alpha and CR values were below 0.50; Items 1, 6, 7, and 11 were excluded from the analysis to improve model fit values. The psychological ownership scale ultimately consisted of 9 items and three dimensions.

#### Utrech work engagement scale

Item 6 of the Urtecht work engagement scale, which consists of six items, was excluded from the analysis in order to improve compliance values, and, finally, the scale was formed as one dimensional with five items.

### Findings related to hypothesis testing

After the verification of the measurement model, the research hypotheses were tested on the implicit variable structural model. First of all, in order to test the H1 (GHRM → work engagement) hypothesis, which is graphically shown in Figure 3, the implicit variable structural model, in which work engagement is exogenous and GHRM is endogenous, was tested. According to SEM results, it was determined that GHRM predicted work engagement behavior (β = 0.3; *p* < 0.01). According to this result, H1 was supported.

**Figure 3:** Path analysis. JD, Job design; SETR, Selection and training; PER, Performance; PAY, Wage management; GHRM, Green human resources management; WE, Work engagement.

GHRM includes four sub-dimensions: job design, selection and training, performance management, and compensation and wage management. A separate model was created to see the effects of GHRM sub-dimensions on work engagement. The fit values of the model are within acceptable limits (*X*^2^*/df* = 1.910, *CFI* = 0.971, *SRMR* = 0.038, and *RMSEA* = 0.060). According to the results of the analysis, it was determined that none of the sub-dimensions alone had a significant effect on the work engagement behavior. Job design (β = 0.28; *p* > 0.05), selection and training (β = 0.18, *p* > 0.05), wages management (β = −0.22, *p* > 0.05).

In order to test the other hypotheses of the research, a separate model was created in which psychological ownership is the mediating variable (Figure 4). According to the mediated structural model analysis results, it was seen that GHRM predicted psychological ownership (β = 0.4; *p* < 0.01). In this case, H2 was supported. Similarly, the effect of the mediating variable, psychological ownership, on work engagement was found to be significant (β = 0.80; *p* < 0.01). In this case, H3 was supported. With the inclusion of the mediator variable, psychological ownership, in the model, the coefficient from GHRM variable to work engagement behavior became meaningless (β = −0.02; *p* > 0.05). Psychological ownership, along with GHRM, explains 62% of the change in work engagement behavior. The indices obtained as a result of the path analysis were within acceptable threshold values in the literature, indicating that the model was compatible with the data [*X*^2^ (425, *N* = 250) = 843.684; *p* > 0.01; *X*^2^/df = 1.985; *CFI* = 0.945; *RMSEA* = 0.063; *SRMR* = 0.063]. The results of the hypothesis tests are shown in Table 4.

**Figure 4:** The structural model with a mediator variable.

**Table 4:** The structural model and hypothesis testing.

	**Output variables**			
	**Psychological ownership**		**Work engagement**	
	**β**	**SE**	**β**	**SE**
GHRM (path)	-	-	0.34^***^	0.44
*R^2^*	-	-	0.12	
GRHM (a path)	0.45^***^	0.040	-	
*R^2^*	0.20		-	
GHRM (c' path)	-		−0.02^***^	−0.013
Psychological Ownerhip (b path)	-		0.80^***^	0.966
*R^2^*	-		0.62	
Indirect effect	-		0.356, (0.206, 0.540)

*** p < 0.001. SE, Standard error; values in parentheses are lower and upper confidence intervals. Bootstrap resampling = 5,000.

GHRM includes four sub-dimensions: job design, selection and training, performance, and payment. To see the effect of sub-dimensions on work engagement, which is an exogenous variable, four different path diagrams were created and tested. According to the results of the analysis, it was observed that all of the GHRM sub-dimensions significantly affected the work engagement behavior. Path analysis and model fit values for GHRM sub-dimensions and the work engagement variable are shown in Table 5.

**Table 5:** GHRM sub-dimensions–work engagement path analysis values.

**Construct**	**β**	**SE**	**Model fit values**
Job design	0.36^*^	0.041	X^2^/df = 1.004, CFI = 1.000, SRMR = 0.039, RMSEA = 0.004
Selection and training	0.35^*^	0.039	X^2^/df = 2.373, CFI = 0.978, SRMR = 0.036, RMSEA = 0.074
Performance	0.29^*^	0.040	X^2^/df = 1.075, CFI = 0.999, SRMR = 0.032, RMSEA = 0.017
Wage management	18^*^	0.041	X^2^/df = 1.622, CFI = 0.990, SRMR = 0.039, RMSEA = 0.050

* p < 0.01. Standardized values are reported.

According to the analysis results, the job design has the highest effect on the work engagement behavior. The effect of the wage management on the work engagement behavior is less than the other dimensions.

The effects of the sub-dimensions of the internal variable GHRM on the mediating variable psychological ownership are shown in Table 6. It is seen that all of the GHRM sub-dimensions have a significant effect on the psychological ownership variable. However, the SRMR values of selection and training, performance, and wage management dimensions are outside the acceptable limits. It is seen that the job design dimension among the GHRM sub-dimensions has the highest effect.

**Table 6:** GHRM sub-dimensions–psychological ownership path analaysis values.

**Construct**	**β**	**SE**	**Model fit values**
Job design	0.48^*^	0.037	X^2^/df = 2.584, CFI = 0.957, SRMR = 0.039, RMSEA = 0.079
Selection and trainig	0.42^*^	0.035	X2/df =1.890, CFI = 0.973 SRMR = 0.010, RMSEA = 0.060
Performance	0.33^*^	0.360	X^2^/df = 2.714, CFI = 0.952, SRMR = 0.011, RMSEA = 0.083
Wage management	0.25^*^	0.035	X^2^/df = 1.890, CFI = 0.973 SRMR = 0.010, RMSEA = 0.060

* p < 0.01. Standardized values are reported.

The effects of the mediating variable psychological ownership sub-dimensions on the exogenous variable work engagement are shown in Table 7. All three sub-dimensions of psychological ownership have a significant effect on work engagement behavior. The effect of the internal responsibility dimension is higher than the other dimensions. The *RMSEA* value of the protective focus size is outside the acceptable limits.

**Table 7:** Psychological ownership sub-dimensions path analaysis values.

**Construct**	**β**	**SE**	**Model fit values**
Self identitiy	0.59^*^	0.056	X^2^/df = 2.555, CFI = 0.973, SRMR = 0.053, RMSEA = 0.079
Protective focus	0.42^*^	0.035	X2/df = 1.641, CFI = 0.989 SRMR = 0.054, RMSEA = 0.106
Internal responsibility	0.70^*^	0.140	X2/df = 3.821, CFI = 0.966 SRMR = 0.065, RMSEA = 0.051

* p < 0.01. Standardized values are reported.

The path analysis based on the bootstrap method was conducted to test whether psychological ownership has a mediating role in the relationship between GHRM and work engagement behavior. It is claimed that the Bootstrap method gives more reliable results than the traditional method of Baron and Kenny (1986) and the Sobel test (Gürbüz, 2019). About 5,000 resampling options were preferred in the mediation effect analyses made with the bootstrap technique. In the mediation effect analyses performed with the bootstrap technique, the 95% confidence interval (CI) value obtained as a result of the analysis should not contain the zero (0) value in order to support the research hypothesis (Gürbüz, 2019). According to the Bootstrap results, the indirect effect of GHRM on the mediation of psychological ownership was found to be significant [β = 0.356, 95% CI (0.206, 0.540)]. These results show that the psychological ownership variable has a mediating effect on the relationship between GHRM and work engagement behavior; in which case, H4 was supported (see Figures 4, 5).

**Figure 5:** The conceptual model of the research.

The conceptual model of the research is shown in Figure 5.

Psychological ownership, which was used as a mediator variable in this study, includes three sub-dimensions: self-identity, personal focus, and internal response. Table 8 shows the mediation analyses regarding the sub-dimensions of the psychological ownership variable. Mediation analyses of sub-dimensions were performed using Model 4 in Hayes Macro.

**Table 8:** Psychological ownership sub-dimensions mediation analyses results.

**Path**	**Effect**	**B**	**BootSE**	**BootLLCI**	**BooTULCI**	**Effect**
GHRM → SI → WE	Direct effect	0.17	0.04	0.0953	0.2433	
	Indirect effect	0.02	0.01	0.0026	0.0497	Yes
GHRM s → PF → WE	Direct effect	0.15	0.03	0.0852	0.3225	
	Indirect effect	0.1439	0.0270	0.0943	0.1992	Yes
GHRM → IR → WE	Direct effect	0.10	0.03	0.0481	1.1353	
	Indirect effect	0.09	0.02	0.0481	0.1353	Yes

BootSE, Bootstrap Standart Error; BootLLCI, Bootstrap %95 confidence l interval lower level; BootULCI, Bootstrap %95 confidence interval upper level. 5,000 Boostrtap is used. GHRM, Green human resources management; SI, Self-identity; WE, Work engagement; PF, Personal focus; IR, Internal responsibility.

According to the results of the analysis, it shows that all sub-dimensions of the psychological ownership variable have a significant mediating effect on the relationship between GHRM and work engagement.

## Discussion

Incorporating corporate environmental sensitiveness into human resources practices is explained as GHRM (Nawangsari and Sutawidjaya, 2019). The GHRM encompasses systems, policies, and practices necessary for developing a socially responsible, resource-efficient, and environmentally sensitive workplace (Waqas et al., 2021). Hence, embracing GHRM practices has become a critic strategy for those companies wherein human resources play an active part in becoming environmentally sensitive (Adriana et al., 2020). In relation to that, GHRM can nurture supporters across employees that are willing to contribute to environment (Khan et al., 2022). In this study, we assumed that being in an environment-friendly atmosphere caused by GHRM will create positive attitudes on the part of employees nourishing their sense of ownership, which will mediate the relationship between GHRM and employees' work engagement.

In this study, first of all, we wanted to test the direct positive effect of GHRM on work engagement levels of employees, and the results revealed that all dimensions of GHRM have a positive effect on work engagement. Our findings are parallel with previous studies showing the direct effect of GHRM on work engagement of employees (Sokro et al., 2020; Bhutto et al., 2021; Waqas et al., 2021). Our results revealed that the job design has the highest effect on the work engagement behavior, whereas the effect of the wage management dimension is the least. These results are parallel with the previous studies on HRM's (a classic form of HRM rather than GHRM) effect on work engagement, in the points that job design is very effective on work engagement and acts as a motivator (Letona-Ibañez et al., 2021; Shang, 2022), but wage management has a rather minor effect (Londa and Permatasari, 2021; Good et al., 2022) since wage is considered as a hygiene factor rather than a motivator.

Moreover, GHRM interventions can encourage employees to take green initiative and engage in green proactive behavior, which is considered as an individual investment according to conservation of resources theory (Jermsittiparsert et al., 2019; Hameed et al., 2022). Without a doubt, companies encouraging their employees to become a part of green initiatives make them feel more identified with their organizations and develop high levels of psychological ownership, owing to their efforts and investments on green issues (Liu et al., 2012). As Curcuruto and Griffin (2018) suggest, prosocial and proactive attitudes of organizations contribute to greater social identification on the part of employees, which can be considered as a source of psychological ownership. So, in this study, it is assumed that GHRM has the capacity to boost employees' feelings of psychological ownership. In the related analysis, it is revealed that GHRM has a positive effect on Psychological Ownership, and job design dimension is the sub-dimension having the highest positive effect. This is mostly because of the strong effect of work structure on psychological ownership (Pierce et al., 2004). Actually, this is the first study revealing the positive effect of GHRM practices on enhancing the psychological ownership of employees. Although not exactly the same model, there are studies showing the positive effect of similar green management approaches on psychological ownership. For instance, Chang's et al. (2020) study resembles our study in the point that it revealed the positive effect of Green Shared Vision on employees' feelings of psychological ownership. Our results are also parallel with the previous studies revealing this positive impact of psychological ownership on work engagement (Wang et al., 2019; Chai et al., 2020) and with studies suggesting that it prevents intention to quit (Su et al., 2021).

Moreover, we also tested whether Psychological Ownership has a positive effect on work engagement. Results revealed that all subdimensions of Psychological Ownership positively affect work engagement. Our results were in parallel with the previous studies, revealing this positive effect on work engagement levels of employees (Khan and Gul, 2021; Nurtjahjani et al., 2021). In this study, we also tested whether psychological ownership acts as a mediator in the relationship between GHRM and work engagement. Results revealed that psychological ownership has a mediator effect on the relationship between GHRM and work engagement with all its sub-dimensions. Our results are parallel with those studies conducted by Gim et al. (2021), revealing the positive indirect effect of GHRM on work engagement through HRM performance attributions as a mediator in the point that, in our study, the effect of GHRM is also ended up to be an indirect effect on work engagement, which occurs through Psychological Ownership. This study is unique in revealing the effect of sense of Ownership in boosting work engagement by GHRM, thus contibutes to both sustainability literature and GHRM literature. Owing to this study, we could emphasize the significance of using GHRM for creating greater sense of ownership and engagement and utilizing GHRM as a motivator for encouraging people to engage their organizations.

## Conclusion

In this study, the effects of GHRM on psychological ownership perceptions and work engagement levels of employees have been examined and the possible mediator effect of psychological ownership has been tested. In the study, GHRM has been examined with four sub-dimensions: green job design, green selection, green education and development, green performance appraisal, and green wage management. A significant and positive relationship was found between all sub-dimensions of this GHRM (green job design, green selection and training, green performance appraisal, and green wage management) and work engagement levels of employees; hence, H1 hypothesis is accepted, which makes us think that, when organizations engage in environmentally friendly human resources practices, their employees feel satisfied and develop greater work engagement. According to the related analysis, job design is the most effective dimension, whereas wage management has the lowest effect. This may be resulting from the fact that green wage management may be creating disadvantages for some employees, and they may be losing money. Anyway in the related literature, wage management is associated with hygiene factors that neutralize its effect as a motivator (Good, Hughes and Wang).

Furthermore, it was revealed that all four dimensions under GHRM have a statistically significant and positive relationship with psychological ownership. Thus, H2 hypothesis is also accepted. Although all dimensions positively affected the psychological ownership, the positive effect of GHRM on Psychological Ownership has mostly come about through the positive effect of job design.

Moreover, in H3, we tested the possible positive effect of psychological ownership on work engagement. Results revealed that all three sub-dimensions of psychological ownership have a significant effect on work engagement behavior. The effect of the internal responsibility dimension is higher than the other dimensions. So H3 is also accepted. This was an expected result since, from the extant literature, we know that the psychological ownership construct is an important antecedent of work engagement (Ugwu and Amazue, 2014; Wang et al., 2019).

Our expectations regarding the mediation effect have also been confirmed. It has been revealed that psychological ownership has a positive mediation effect between work engagement and GHRM applications, so H4 is also accepted. This is a noteworthy and valuable contribution to the literature. This study makes a great contribution to the literature in order to show how GHRM affects the sense of ownership of employees' organizations and how commitment can be increased through this effect. Hence, creating the sense of ownership should be considered as a tool for increasing the positive effect of GHRM on the engagement level of employees. Without a doubt, what makes this study unique in the point is the fact that it revealed the mediating effect of psychological ownership in the relationship between GHRM and work engagement. Thus, this study is important for confirming the importance of GHRM as a tool for boosting engagement and revealing the significance of psychological ownership in more engaged employees.

### Managerial implications

Actually, companies embracing GHRM can easily build a positive organizational image and contributes to work engagement of their employees (Nawangsari and Sutawidjaya, 2019). In this sense, GHRM can be adopted as a mechanism that strengthens both engagement and sense of psychological ownership. Hence, this study is noteworthy in the point that it showed that GHRM, as an intrinsic motivation tool, affects psychological ownership and increases work engagement through this effect. The fact that this study is the first study revealing the significance of GHRM practices on work engagement levels of Turkish employees, we believe that this is an encouraging and challenging study for Turkish employers who are mostly hesitant about using GHRM as a motivational tool. According to our results, the effects of job design and training and development dimensions on work engagement behavior are higher than performance and payment dimensions. This result can be evaluated as an indication that businesses should seriously consider GHRM applications during the job design and selection phase. If we put the sentence in reverse, businesses that do not show the necessary care in the job design and selection stages in the GHRM application may not be successful in influencing the work engagement behavior of their employees with only performance and wage management.

### Further studies and limitations

Owing to this study, the effect of GHRM on psychological ownership has been illuminated. This is the first study revealing the positive effect of GHRM on psychological ownership, and it is also the first study revealing the mediator effect of psychological ownership in the relationship between GHRM and work engagement. The fact that the sample of this study is white-collar employees working in production companies in Turkey creates the biggest limitation on the generalizability of the study. In order to make the study more generalizable, wider geographies and greater number sectors can be included in the sample. The model can also be tested in cross-cultural studies or longitudinal studies. Moreover, a moderator variable can beadded to the model, making the model more comprehensive. For instance, testing the moderator effect of employee proenvironmental attitude can be useful. Future research may also point out whether the effect of the independent variables in different generations of respondents is valid. Furthermore, different dependent variables, such as corporate organizational citizenship, job satisfaction or job performance, can be tested.

## Data availability statement

The raw data supporting the conclusions of this article will be made available by the authors, without undue reservation.

## Ethics statement

Ethical review and approval was not required for the study on human participants in accordance with the local legislation and institutional requirements. The patients/participants provided their written informed consent to participate in this study.

## Author contributions

Both authors listed have made a substantial, direct, and intellectual contribution to the work and approved it for publication.

## Conflict of interest

The authors declare that the research was conducted in the absence of any commercial or financial relationships that could be construed as a potential conflict of interest.

## Publisher's note

All claims expressed in this article are solely those of the authors and do not necessarily represent those of their affiliated organizations, or those of the publisher, the editors and the reviewers. Any product that may be evaluated in this article, or claim that may be made by its manufacturer, is not guaranteed or endorsed by the publisher.
